# Effect of Health Education Combined with Dietary Guidance on Nutritional Indicator, Immune Level, and Quality of Life of Patients with Pulmonary Tuberculosis

This article has been retracted.

**DOI:** 10.1155/2021/9463577

**Published:** 2021-09-29

**Authors:** Baojuan Hu, Guoxia Ren, Lin Zhao

**Affiliations:** Xi'an Chest Hospital, Xi'an 710100, China

## Abstract

**Objective:**

To investigate the effects of health education combined with dietary guidance on nutritional indicators, immune level, and quality of life of patients with pulmonary tuberculosis.

**Method:**

A total of 123 patients with pulmonary tuberculosis who were hospitalized to our hospital between October 2019 and October 2020 were chosen for the study and were separated into 60 control cases and 63 observation cases based on the ward they were assigned to. Patients in the two groups were compared in terms of nutritional risk, nutritional indicator levels in serum, immunological function, treatment compliance, sputum culture conversion rate, and quality of life.

**Result:**

With the prolongation of patients' illness, the total NRS 2002 score gradually increased in both groups and the total NRS 2002 score of patients in the control group was higher than that of patients in the observation group at the same time point after discharge. The difference between the total NRS 2002 score of patients in both groups was significant at 3 and 6 months after discharge. After the intervention, the Hb, ALB, CD4+, and CD4+/CD8+ levels of patients in both groups were higher than those at the time of admission, and the CD8+ levels were lower than those at the time of admission. At 6 months after discharge, the Hb, ALB, CD4+, and CD4+/CD8+ levels of patients in the observation group were significantly higher than those in the control group, and the CD8+ levels were significantly lower than those in the control group. The treatment compliance rate of patients in the observation group (96.83%) was significantly higher than that of the control group (75%), and the negative sputum culture transfer rate (85.71%) was significantly higher than that in the control group (60%). The overall quality of life scores of patients in the observation group was significantly higher than that in the control group.

**Conclusion:**

Health education combined with dietary guidance for patients with pulmonary tuberculosis can deepen patients' understanding of disease and nutritional knowledge, improve treatment compliance, improve their nutritional status, enhance their immune function, accelerate sputum bacterial conversion, enhance treatment effect, and improve their quality of life.

## 1. Preface

Pulmonary tuberculosis (PTB) is a chronic infectious disease of the respiratory tract and is an airborne disease caused by *Mycobacterium tuberculosis* (MTB) [1]. According to a report on the global TB situation published by WHO in 2019, about 10 million people suffered from PTB worldwide in 2018, and China has become one of the 22 high-burden TB countries identified by WHO, with 14.3% of patients worldwide, ranking third in the world [2].

Immunocompromised and weak people are vulnerable to PTB, and PTB patients commonly suffer from dyspnea, cough, and afternoon hypothermia. Prolonged hypothermia promotes catabolism in the body, resulting in poor absorption of gastrointestinal functions and a loss of hunger, which leads to varying degrees of malnutrition. Studies confirmed that the onset of PTB in 32%-62% of patients with PTB is due to malnutrition [3]. At the same time, malnutrition can lead to dysfunction of body tissues and organs, which can especially reduce cellular immune function, thus contributing to the development of PTB [4].

Currently, the incidence of PTB has been better controlled through the efforts of governments and people, but the high relapse rate of PTB is still a major challenge in PTB control. Multidrug-resistant tuberculosis (MDR-TB) and extensively drug-resistant tuberculosis (XDR-TB) patients have poor treatment results, with just 54% of patients obtaining favorable outcomes. [5].

Bestrashniy et al. and Mirsaeidi et al. showed that treatment compliance is a protective factor for PTB, and patients with high treatment compliance had a relapse rate of only 1.1%, while patients with low treatment compliance had a relapse rate of 50% [6, 7]. Since PTB is an infectious disease, low patient compliance to treatment not only reduces the effectiveness of treatment but also affects the health of others and increases the burden of disease on society as a whole. In the 1990s, WHO developed the DOTS strategy, including five aspects of government commitment, free drug supply, systematic monitoring, patient identification, and direct observation of patients taking medication by medical staff, a project that is aimed at enhancing PTB by using a better patient management approach and enhancing patient adherence to therapy, increasing illness cure rates, and improving disease control [8, 9].

The purpose of this study is to analyze the effects of this intervention on the nutritional indicator, immune level, and quality of life of patients with pulmonary tuberculosis (PTB) by using health education combined with dietary guidance, in order to offer a theoretical foundation for enhancing PTB patients' compliance and treatment results. The following are the specifics.

## 2. Information and Method

### 2.1. General Information

One hundred and twenty-three cases of pulmonary tuberculosis patients admitted to our hospital from October 2019 to October 2020 were selected as the study subjects and grouped according to the ward to which the patients belonged, with 60 patients from the first ward as the control group and 63 patients from the second ward as the observation group. All patients met the diagnostic criteria of the Diagnosis of Tuberculosis in the Health Industry Standard of the People's Republic of China implemented in China in May 2018, and the sputum culture was positive for binding bacilli.

Inclusion criteria were as follows: (1) the age of patients is between 18 and 65 years, (2) patients have consciousness and normal intelligence, (3) there are no concurrent heart, liver, renal, or other chronic illnesses in the patients, and (4) patients freely participated in this research after signing an informed consent form.

Exclusion criteria were as follows: (1) patients have severe anemia, (2) patients have severe impairment of major organ function, (3) patients have cognitive impairment, (4) patients are in pregnancy or lactation, and (5) patients have poor treatment compliance and do not accept the survey during the follow-up.

This research topic has been reviewed and approved by the ethics committee of our hospital.

### 2.2. Intervention Method

Patients in both groups were given antituberculosis drugs according to their condition and were treated and observed for 6 months. Both groups of patients returned their current health status through WeChat or telephone.

Patients in the control group received regular care, and nursing personnel provided medication and food advice to patients and their families based on their own expertise and clinical experience.

The following is a list of health education and nutrition advice provided to patients in the observation group.

### 2.3. Establishment of Professional Nursing Team

A professional nursing team was formed by 2 doctors, 1 head nurse, 3 charge nurses, 8 bedside nurses, 1 nutritionist, and 1 psychological counselor. The division of responsibilities is clearly defined, and the patient's demographic data, disease condition, and nutritional status are assessed by means of questionnaires to lay the foundation for carrying out follow-up care.

### 2.4. Health Education

After patients are admitted to the hospital, the nursing staff introduce patients to the hospital, working and resting hours, etc. to help patients and their families adapt to the hospital environment. Regularly organize expert lectures, in which the experienced medical and nursing staff introduce patients and their families to knowledge about the disease, side effects of antituberculosis drug use, how to prevent adverse drug reactions, etc., so that patients may properly assess the illness, encourage patients to establish regular medication habits, alleviate patients' worries, and increase their confidence in their ability to overcome the disease. We invite cured patients to share their experiences, communicate with patients and their families, understand patients' confusion in the treatment process, help patients analyze the causes and solve difficulties, use words that patients can understand in the communication process, and communicate sincerely to increase patients' trust in medical staff. For patients who have poor treatment compliance during treatment, we will understand the reasons in time and intervene by dedicated personnel to prevent patients from shedding.

### 2.5. Dietary Guidance

A nutritional risk assessment was conducted based on the patient's nutritional status, and an individualized diet plan was developed for the patient. Patients are advised to consume more high-quality, high-protein foods, such as lean meat, eggs and freshwater fish, more fresh vegetables, and foods rich in B vitamins, prohibit the use of spicy and stimulating foods and drinks containing caffeine, and quit smoking and limit alcohol. A Nutrition Guidance Manual and a propaganda video were developed to educate patients about the link between PTB's nutritional status and illness development, as well as the significance of nutritional treatments for patients.

### 2.6. Observation Indicators and Evaluation Criteria

#### 2.6.1. Nutritional Risk Screening

In 2003, the European Society of Clinical Nutrition and Metabolism first proposed the NRS 2002 Nutrition Risk Screening Scale, which was developed based on 128 clinical studies focusing on patients' nutritional status and disease severity and is very effective in predicting the risk of malnutrition and the outcome of nutritional therapy with good reliability and validity [10]. The total NRS 2002 score is the sum of the disease severity, and the sum of three component scores reduced nutritional status and age status, with a maximum score of 7 and a minimum score of 1. The higher the patient's score, the greater the likelihood of nutritional risk, which is usually defined as the presence of malnutrition risk with a total NRS 2002 score ≥ 3. NRS 2002 nutritional risk screening was performed at the time of admission, 1 month, 3 months, and 6 months after discharge to evaluate the nutritional status of the patients.

### 2.7. Nutritional Indicator Level

To assess Hb and ALB levels at the time of admission and 6 months after release, fasting venous blood was taken early in the morning and serum was extracted by centrifugation at 3500 r/min for 10 minutes. Patients were considered anemic when Hb was less than 120 g/L and hypoproteinemic when ALB was less than 35 g/L [11].

### 2.8. Immune Function

At the time of admission and at the time of return for review at 6 months after discharge, 5 mL of fasting peripheral venous blood was drawn from patients in the early morning in heparin anticoagulation tubes, CD4+ and CD8+ were determined by flow cytometry, and CD4+/CD8+ was calculated.

### 2.9. Treatment Compliance

At 6 months after discharge from the hospital, patients' compliance to treatment was evaluated by using an in-hospital developed treatment compliance questionnaire, which covered four aspects: taking medication on time and in the right amount, eating selectively according to the dietary guidance program, conducting regular review, and consciously cooperating with the doctor's treatment plan, and was divided into three dimensions: nonadherence, adherence, and very adherence. Patients who were completely able to follow the doctor's medication and selective diet prescriptions were classified as fully compliant; patients who were only partly able to follow the doctor's medication and selective diet prescriptions were classified as somewhat compliant. Patients who were not able to follow the doctor's prescriptions for medication and selective diet for more than half of the observation period were evaluated as poorly compliant.

(1) $$\begin{array}{c} Treatment\;compliance\;rate=\frac{number\;\text{of }full\;compliance\;cases+number\;\text{of }partial\;compliance\;cases}{total\;number\;\text{of }cases}. \end{array}$$

### 2.10. Negative Sputum Culture

At 6 months after discharge, the patients' sputum was tested for *Mycobacterium tuberculosis* at the time of their follow-up visit, and the rate of sputum culture conversion was calculated to evaluate the effect of the intervention.

### 2.11. Quality of Life

The SF-36 scale was used to evaluate the quality of life of patients, and studies have shown that the SF-36 scale was used to evaluate the quality of life of PTB patients with high reliability and validity [12, 13].

The SF-36 scale contains 8 dimensions of physical functioning, physical role, mental health, emotional role, social functioning, vitality, physical pain, and general health, with a total of 36 items. The raw scores are first calculated to obtain the raw scores, and the scores are transformed according to a standardized formula, with higher scores representing better quality of life.

(2) $$\begin{array}{c} Conversion\;score=\frac{item\;maximum\;score-item\;minimum\;score}{item\;possible\;score\;range}*100. \end{array}$$

### 2.12. Statistical Method

Excel was used for data entry, and SPSS 25.0 software was used for data analysis. The measurement data were expressed as the description of $\bar{x}\pm s$. The count data were represented as a percentage description, and the independent *t*-test was employed to compare groups. *P* < 0.05 was considered to have a statistically significant difference.

## 3. Result

### 3.1. Comparison of the Differences in General Clinical Indicators between the Two Groups of Patients

The comparison revealed that the general clinical indicators such as gender, age, duration of disease, and type of tuberculosis in the control and observation groups were not statistically significant (*P* > 0.05) and were comparable (Table 1).

### 3.2. Comparative Analysis of Nutritional Risk Screening before and after the Intervention

The difference in the total NRS 2002 score between the two groups of patients at the time of admission was not significant (*P* > 0.05), and with the prolongation of the patients' illness, the total NRS 2002 score gradually increased in both groups and the total NRS 2002 score of patients in the control group was higher than that of patients in the observation group at the same time point after discharge, and the difference in the total NRS 2002 score between the two groups of patients at 3 and 6 months after discharge was significant (*P* < 0.05) (Figure 1).

### 3.3. Comparative Analysis of Nutritional Indicator Level before and after the Intervention

Through the intervention, the serum levels of Hb and ALB in both groups increased compared with those at the time of admission, and at 6 months postdischarge monitoring, the serum levels of Hb and ALB in the two groups differed significantly, and the serum levels of Hb and ALB in the patients in the observation group were significantly higher than those in the control group (Figure 2).

### 3.4. Comparative Analysis of Cellular Immune Function before and after Intervention

Through the intervention, the CD4+ and CD4+/CD8+ levels increased and CD8+ levels decreased in both groups compared with the admission, and at 6 months postdischarge monitoring, the CD4+, CD8+, and CD4+/CD8+ levels differed significantly between the two groups, with the CD4+ and CD4+/CD8+ levels significantly higher in the observation group than in the control group and the CD8+ levels significantly lower than that in the control group (Figure 3).

### 3.5. Comparative Analysis of Treatment Compliance after Intervention

According to the evaluation of patients' compliance with treatment according to the treatment compliance questionnaire, patients in the observation group achieved 74.60% complete compliance and 22.22% partial compliance, with a treatment compliance rate of 96.83% significantly higher than that of 75% in the control group (Figure 4).

### 3.6. Comparative Analysis of Sputum Culture Conversion after Intervention

Six months after discharge, the number of patients in the observation group with negative sputum culture reached 54 cases, and the negative sputum culture transfer was 85.71%, while the number of patients in the control group with negative sputum culture reached 36 cases and the negative sputum culture transfer reached 60%; the rate of sputum culture transfer in the observation group was significantly higher than that in the control group (Table 2).

### 3.7. Comparative Analysis of Quality of Life before and after Intervention

The SF-36 scale was used to assess the quality of life of patients in both groups. The difference between the total quality of life scores of the two groups at admission was not significant (*P* > 0.05), and through the intervention, at 6 months after discharge, the total quality of life scores of patients in both groups was higher than that at admission and the total quality of life scores of patients in the observation group was significantly higher than that of patients in the control group (*P* < 0.05) (Figure 5).

## 4. Discussion

PTB is an important public health safety issue in China, and the disease is a chronic respiratory infectious disease with a treatment process divided into two phases, an intensive treatment phase and a consolidation phase [14]. The treatment process for PTB is long, the intense treatment phase lasts just 1-2 months (up to 3 months for drug-resistant patients), and the rest of the time is spent at home consolidating the therapy [15]. The successful recovery of the patient is related to the patient's awareness of the disease and compliance with medication and diet during treatment.

Lange et al. showed that 4.6% of PTB patients worldwide are caused by multidrug-resistant TB, and in countries such as Kazakhstan and Ukraine, this percentage even exceeds 25%, and patients with multidrug-resistant TB take longer to treat [16]. Several studies domestically and internationally have shown that one of the main reasons for the emergence of drug-resistant TB is due to irregular treatment of patients and low compliance with medication [17, 18]. For the development of medication resistance, it is thus critical to ensure that patients have a thorough understanding of the illness and that they adhere to their treatment regimens.

Studies have shown that nutritional risk is associated with clinical outcomes of patients. Nutritional risk in patients increases the risk of complications, leads to poor clinical outcomes, and can even increase mortality [19, 20]. In PTB, as a wasting disease, early intervention of dietary guidance to patients can improve the level of nutritional knowledge and draw the attention of patients. Scientific nutritional support can reduce the incidence of adverse reactions and promote the recovery of the disease [21]. Currently, the WHO has recommended nutritional assessment of PTB patients as an integral part of their care [22].

In this study, by using the intervention of health education combined with dietary guidance during the treatment of pulmonary tuberculosis, the results showed that the difference in the total NRS 2002 score between the two groups of patients at the time of admission was not significant (*P* > 0.05). The total NRS 2002 score of patients in both groups gradually increased with the prolongation of the patients' illness, and the total NRS 2002 score of patients in the control group was higher than that of patients in the observation group at the same time point after discharge. The difference between the NRS 2002 total scores of patients in the two groups at 3 and 6 months after discharge was significant (*P* < 0.05), which may be due to the fact that the possibility of nutritional risk of patients is increasing with the increase in patients' treatment time. The observation group, through health education and dietary guidance, was able to provide patients with targeted nutritional support, so that patients could take in the nutrients required by the body through a reasonable diet in daily life, thus significantly reducing the incidence of nutritional risk and playing a positive role in improving the nutritional status of patients. The serum level of Hb and ALB in both groups was higher than that at the time of admission, and the difference between the serum level of Hb and ALB in the two groups was significant when monitored 6 months after discharge. The serum level of Hb and ALB in the observation group was significantly higher than that in the control group (*P* < 0.05), which may be due to the high catabolic rate and serious protein loss after PTB due to the influence of the disease. The rapid growth of tuberculosis bacilli consumes the nutrients required by hematopoietic cells, leading to anemia and other symptoms in patients [23]. For the emergence of medication, it is critical to ensure that patients have a thorough understanding of the illness and that they adhere to their treatment regimens. Patients' serum levels of Hb and ALB were higher than those in the control group after receiving health education and dietary guidance, demonstrating that this intervention can provide patients with the amount of protein required by the organism, increase nutrient absorption efficiency above the metabolic rate, increase the patient's protein reserve, and improve nutritional status. CD4+ cells are helper T cells, and they are resistant to infection, which secrete a variety of cytokines through the Th1-type cellular immune response CD8+ which is the opposite of the CD4+ immune effect; CD8+ suppresses cellular and humoral immunity through immune regulation, high level of CD8+ expression mostly indicates the deterioration of PTB condition, when the balance between CD4+ and CD8+ is disrupted, and the immune function of the body is hindered and vulnerable to pathogenic bacteria [24, 25]. Through the intervention, the CD4+ and CD4+/CD8+ levels increased and CD8+ levels decreased in both groups compared to those at the admission, and at 6 months postdischarge monitoring, the CD4+ and CD4+/CD8+ levels were significantly higher and CD8+ levels were significantly lower in the observation group than in the control group, which may be due to the fact that health education and dietary guidance provided to patients were able to regulate the function of T lymphocyte subpopulations in PTB patients and enhance the immune capacity of the body.

In summary, health education for patients with tuberculosis can enable patients to correctly understand the disease, improve treatment compliance, establish mutual trust with medical and nursing staff through communication, and build confidence in overcoming the disease. Scientific dietary guidance by professionals according to patients' physical condition can improve patients' dietary habits, increase nutrient intake, reduce the incidence of nutritional risks, improve patients' organism immunity to a certain extent, and substantially improve patients' quality of life. Therefore, this approach has the significance of clinical promotion.

## Figures and Tables

**Figure 1:** Comparison of nutritional risk screening between the two groups of patients before and after the intervention. The total NRS 2002 score gradually increased in both groups as the patients' illness progressed, and the total NRS 2002 score of patients in the observation group was significantly lower than that of patients in the control group at 3 and 6 months after discharge (∗ represents *P* < 0.05 between groups after the intervention).

**Figure 2:** Comparison of serum levels of nutritional indicators between the two groups of patients before and after the intervention. Serum levels of Hb and ALB were higher in both groups after the intervention, and at 6 months after discharge, serum levels of Hb and ALB were significantly higher in the observation group than in the control group (∗ represents *P* < 0.05 between groups after the intervention).

**Figure 3:** Comparison of cellular immune function between the two groups before and after intervention. After the intervention, the CD4+ and CD4+/CD8+ levels of patients in both groups were higher than those at the time of admission and the CD8+ levels were lower than those at the time of admission. At 6 months after discharge, patients in the observation group had substantially greater CD4+ and CD4+/CD8+ levels than those in the control group, but CD8+ levels were significantly lower (∗ indicates the intergroup *P* < 0.05).

**Figure 4:** Comparison of treatment compliance between the two groups of patients after the intervention. After the intervention, patients in the observation group (b) achieved 74.60% complete compliance and 22.22% partial compliance, with a treatment compliance rate of 96.83% significantly higher than the treatment compliance rate of 75% for patients in the control group (a).

**Figure 5:** Comparison of total quality of life between the two groups before and after the intervention. The total quality of life scores of patients in both groups increased after the intervention compared with that at admission, and the total quality of life scores of patients in the observation group were significantly higher than that of patients in the control group (∗ represents *P* < 0.05 between groups after the intervention).

**Table 1:** Comparison of general clinical indicators between the two groups ($\bar{x}\pm s$/*n* (%)).

	Control group (*n* = 60)	Observation group (*n* = 63)	*t*/*X*^2^	*P*
Gender			0.011	0.916
Male	32	33		
Female	28	30		
Average age (years)	42.91 ± 7.10	43.21 ± 6.93	0.054	0.975
Duration of disease (years)	2.76 ± 1.23	2.89 ± 1.15	0.173	0.863
Types of tuberculosis			0.333	0.564
Chronic fibrous cavity	45	50		
Tuberculous pleurisy	15	13		

**Table 2:** Comparison of sputum culture conversion between two groups of patients.

Group	Turning cloudy	Not turned negative	Conversion rate (%)
Control group (*n* = 60)	36	24	60
Observation group (*n* = 63)	54	9	85.71
*X* ^2^			10.351
*P*			0.001

## Data Availability

The data used to support the findings of this study are included within the article.
